The article "Role of Antimicrobial Drug in the Development of Potential Therapeutics" was published in 2022. Journal: Evid Based Complement Alternat Med.

# Role of Antimicrobial Drug in the Development of Potential Therapeutics

**DOI:** 10.1155/2022/2500613

**Published:** 2022-05-05

**Authors:** Shilpa Borehalli Mayegowda, Manjula NG, Saad Alghamdi, Banan Atwah, Zain Alhindi, Fahadul Islam

**Affiliations:** ^1^School of Basic and Applied Sciences, Dayananda Sagar University, Bengaluru, Karnataka, India; ^2^Laboratory Medicine Department, Faculty of Applied Medical Sciences, Umm Al-Qura University, Makkah, Saudi Arabia; ^3^Department of Pharmacy, Faculty of Allied Health Sciences, Daffodil International University, Dhaka 1207, Bangladesh

## Abstract

Population of the world run into several health-related emergencies among mankind and humans as it creates a challenge for the evolution of novel drug discoveries. One such can be the emergence of multidrug-resistant (MDR) strains in both hospital and community settings, which have been due to an inappropriate use and inadequate control of antibiotics that has led to the foremost human health concerns with a high impact on the global economy. So far, there has been application of two strategies for the development of anti-infective agents either by classical antibiotics that have been derived for their synthetic analogs with increased efficacy or screening natural compounds along with the synthetic compound libraries for the antimicrobial activities. However, need for newer treatment options for infectious diseases has led research to develop new generation of antimicrobial activity to further lessen the spread of antibiotic resistance. Currently, the principles aim to find novel mode of actions or products to target the specific sites and virulence factors in pathogens by a series of better understanding of physiology and molecular aspects of the microbial resistance, mechanism of infection process, and gene-pathogenicity relationship. The design various novel strategies tends to provide us a path for the development of various antimicrobial therapies that intends to have a broader and wider antimicrobial spectrum that helps to combat MDR strains worldwide. The development of antimicrobial peptides, metabolites derived from plants, microbes, phage-based antimicrobial agents, use of metal nanoparticles, and role of CRISPR have led to an exceptional strategies in designing and developing the next-generation antimicrobials. These novel strategies might help to combat the seriousness of the infection rates and control the health crisis system.

## 1. Introduction

Nature has been a rich source for novel finding of potential therapeutic agents that span millions of microbes. Natural products that have been developed are a potential source of antimicrobials and other important metabolites. Microorganisms have been variedly used for the large-scale production of such compounds and have been successful in treatment alternatives that include diseases such as cancer, infectious diseases, diabetes, diarrhoea, atopic dermatitis, and Crohn's disease. They have been a potential source of natural products that include antioxidants, antimicrobials, vitamins, enzymes, immunosuppressants, and enzymes inhibitors. The dawn of antibiotic era has also given a reality check on the emerging antibiotic resistance strains that are dangerous with a disturbing regulatory resistance pattern. The existence of such pathogens came into recognition only in the last 20 years. The escalating MDR pathogens have entitled the researchers for necessitating the postantibiotic era to help in reducing the mortality rate worldwide. Lack of research in developing the newer antibiotics is one of the key factors that have led to the crisis in medical field and denoted elsewhere [1, 2]. The Centre for Disease and Dynamics, Economics and Policy has well documented on the global status of antibiotics policy for better understanding the resistance patterns and need for newer antimicrobials [3]. From 1940 to 1962, there was a rapid development of antibiotics and it is clinically evident from the documentation that about 20 classes had been specified. But in the later years, only two classes have been identified and have been commercialised. However, recently larger pharmaceutical companies have committed towards the drugs treating lifestyle diseases and also yielding high substantial profits [4]. These industry-based partnerships with the smaller companies, academicians, and scientists have helped further in the significant development of antibiotics and its delivery systems.

The article "Role of Antimicrobial Drug in the Development of Potential Therapeutics" was published in 2022. Journal: Evid Based Complement Alternat Med.

### 1.1. Antibiotics: A Wonder Drug for Treating Infections and Its Resistance

Modern medications and technology have been a boon for helping to achieve various aspects for the treatment options related to infectious diseases. One such important key accomplishment has been the discovery of antibiotics that was a boon for human health. However, their misuse has made a very immoral impact on these pathogens in developing resistance factor for various antimicrobials. Thus, it has further complicated and restricted their use in the long-term and its efficacy too. With the discovery of penicillin, other antimicrobials have been elucidated based on the target sites as well as drug molecule modifications. The cell deaths caused by these antimicrobials on bacterial specific target sites involve the cellular structure, biochemical, and molecular levels. The antibiotics induce the death in the pathogens, which is caused due to the breaks in double-stranded DNA followed by the treatment with DNA gyrase inhibitors [5]; following treatment with rifamycin stops the DNA-dependent RNA synthesis [6]; damage caused by cell wall inhibitors on the cell envelop along with the loss of structural integrity [7]; and protein mistranslation, cellular energetics, and ribosomal binding by the protein synthesis inhibitors [8]. Currently, research has proved the mechanism of cell death is due to the drug-induced stress caused by all classes of antimicrobials [9]. Specific treatment options with lethal concentration of antibiotics produce hydroxyl radicals that are harmful through oxidative damage following cellular death pathway by altering the tricarboxylic acid cycle and iron metabolism [10, 11].

Microorganisms over a period have evolved and adjusted according to the environmental changes with subsequent development with various protective mechanisms for their survival strategies in order to reduce their antibiotic susceptibility. Major of these antimicrobials have been losing their efficacy and potency over a period of time with incautious use. Thus, making them useless for the infectious treatment that was once successfully used to treat them. However, with the introduction of new antibiotic class, it has also led to the expansion of resistance levels and it has been utmost evident with their increasing clinical implication shortly after being bought in the market [12]. The cause of MDR in microbes is due to the mutation factor and by the horizontal gene transfer (HGT) between and within the species [13]. It has been observed that there is a rapid and broadly increased dissemination of antimicrobial resistance genes through HGT, especially in *Enterobacteriaceae* family such as encoding *β*-lactamases that includes extended spectrum *β*-lactamases and the metallo-*β*-lactamases (ESBLs and MBLs, respectively) [14, 15], and it is a serious matter of concern that has reached pandemic proportions in healthcare settings worldwide [16, 17]. These *β-*lactamases acquired pathogens have evolved as MDR strains, thus limiting to help in treating the infectious diseases, and in worst cases, the bacterial resistance to carbapenems has left us with treatment options using older and more toxic drugs like colistin [18].

Nevertheless, hospitals acquired infections are already accompanied with high antibiotic resistance; however, recent years have also witnessed the gradual increase in the community-associated infections too [19]. Furthermore, globalisation has led the bacterial genes to travel faster than before and spreading the MDR strains worldwide. Henceforth, it becomes primary importance to find newer antibiotics to control these MDR strains. To combat issues related to MDR pathogens recently, antimicrobial science and technology have gained advancement and helped to include strategies in antimicrobial discovery, different types of novel antibiotics, and using newer materials as antimicrobials to target the pathogens to be researched for the purpose.

The article "Role of Antimicrobial Drug in the Development of Potential Therapeutics" was published in 2022. Journal: Evid Based Complement Alternat Med.

### 1.2. Bacterial Target Sites That can Help for Newer Antibiotics

*Staphylococcus aureus* and *Bacillus subtilis* encode for the cardiolipin by mutated gene, suggesting that it can be an antibiotic target. A novel antibiotic, teixobactin, prevents the biosynthesis of cell wall by binding the lipid pyrophosphate-sugar motif of lipid II precursor in the peptidoglycan and lipid III in the cell wall of teichoic acid in Gram-positive bacteria (Figure 1). LptD, a specific protein inhibitor, inserts to the lipopolysaccharide in the outer membrane called POL70780 in *Pseudomonas aeruginosa*, which can act as target site [20]. Biosynthetic pathway in *Yersinia pestis and P. aeruginosa* has been elucidated, and by using “Staphylopine,” a tetrapeptide isolated from *S. aureus* binds to cobalt, zinc, nickel, and iron can be used to treat with broad-spectrum antibiotics [21]. Peptidoglycan biosynthesis requires lysine and L,L-diaminopimelate aminotransferase (DapL) pathway that leads to the synthesis of lysine, which identified recently in pathogens such as *Chlamydia, Leptospira, and Treponema* [22]. The distribution of enzyme among these pathogens also has potential DapL inhibitors that can act as a narrow-spectrum antibiotic [23]. *Helicobacter pylori and Mycobacterium tuberculosis* are regarded as high MDR pathogens that produce enzymes like shikimate kinase and type II dehyroquinase, which have significant roles in shikimate pathway, and inhibitors for these enzymes are being researched and are under development [24]. Many of the proteins such as TrpB, TrpC, and TrpE for tryptophan biosynthetic pathway in *M. tuberculosis* are studied for their inhibitory molecules that are facilitated by X-ray diffraction structures in Tuberculosis Structural Genomics Consortium (TBSGC) [25, 26]. *M. tuberculosis* has shown promising results in Lassomycin, a peptide produced by *Lentsea spp,* and actinomycetes that inhibit an essential protease enzyme, thus killing both the growing and dormant cells [27]. A study also reveals the mechanism of antibiotic action in food items such as raffinose in ginger that effectively helps to inhibit *P. aeruginosa* biofilm, wherein the intracellular levels of cyclic-di-GMP are decreased to induce motile planktonic cells [28].

## 2. Sources of Antimicrobial Agents

### 2.1. Antimicrobial from Plant Origin

Essential oils derived from the plants are efficient, which depends on their chemical structure, particularly with the hydrophilic functional groups that they possess such as the hydroxyl groups [29]. The compounds of these naturally occurring essential oils (EOs) are the volatile secondary metabolites that are derived from different parts of the plants [30, 31]. The components of essential oils are had been variously studied and have different characteristics like the polypeptides, phenols, tannins, polyphenols, quinones, terpenoids, flavones, lectins, and alkaloids. These metabolites exhibit varied potential activities such as anti-inflammatory, antibacterial, antiviral, antiparasitic, anticancer, antiseptic, antiallergic, and antioxidant. The components of EOs of terpenes such as menthol, geraniol, carvacrol, and thymol have proved with higher antimicrobial activities (Table 1). Relatively, with respect to the individual metabolites, the multiple compounds or the finished EOs are highly efficient and have greater antimicrobial activities [32]. A phenolic compound, Eugenol, is volatile in nature and mainly extracted component from cloves with 70–90% and is accountable for the characteristic clove aroma. It plays a significant role in the oral hygiene and has been used in dental and oral-related preparations, employed as a flavouring agent, sensitiser, irritant, and also as anaesthetic forms. Dental materials adsorbed with eugenol have been employed in clinical dentistry, and it is highly effective against Gram-negative bacteria such as *E. coli, Clostridium botulinum, Shigella, Salmonella,* and *Listeria monocytogenes* [33].

The article "Role of Antimicrobial Drug in the Development of Potential Therapeutics" was published in 2022. Journal: Evid Based Complement Alternat Med.

One of the foremost important EOs is thymol that is derived from the thymes in the form of monoterpene phenol. It exhibits various activities that include antioxidant, anti-inflammatory, antibacterial, antifungal, antiviral, and anti-immunomodulatory effects. It is highly effective, acts by damaging the membrane integrity, change in pH, homeostasis, and equilibrium of inorganic ions against *Salmonella and Staphylococcus spp.* [29]. Another phenolic compound derived from vanilla pods has tremendous industrial applications in food, beverages, perfumes, pharmaceuticals, and also used as nutraceuticals [34]. It has inhibitory effects on the food-spoiling microbes, several fungi, and various pathogens such as *Escherichia, Klebsiella, Salmonella, Bacillus, Serratia, Staphylococcus,* and *Listeria* (Table 1) [35]. A phenolic compound caffeic acid (3, 4-dihydroxycinnamic acid) is derived from the hydroxycinnamic acid, which has some of the exciting biological properties that include fungicide, antibacterial, and antioxidant. Its antibacterial activity has been effective against different pathogens such as *S. epidermidis, S aureus, and K. pneumoniae.*

The article "Role of Antimicrobial Drug in the Development of Potential Therapeutics" was published in 2022. Journal: Evid Based Complement Alternat Med.

The phenolic metabolites, coumarins, are fabricated from benzene and alpha pyrone ring that are fused together. Even though they have a greater activity against fungi, it also proved well that they can control bacteria [36, 37]. Tannin is a polymeric phenolic substance that may be used to tanning leather and to precipitate gelatin from a solution with astringency. Ellagitannins are also a potent compound that can be used in the medical field. Among several tannins, ellagitannins are present in different parts of the plants and have been an excellent source for inhibiting antimicrobial activities against *E coli, S aureus, Salmonella typhimurium, B. subtilis, Shigella sonnei,* MDR *E. coli, K. pneumonia,* and *C. albicans.* These metabolites bind to the cell wall of the bacteria and thus inhibit their growth [38] (Figure 1).

Nonalcoholic beverages are widely used and consumed by humans with an estimate of over two-third of the population as it acts as mild stimulant, refreshing, and medicinal properties. Tea (*Camellia sinensis*) is one among the foremost popular nonalcoholic beverages loaded with polyphenols and epigallocatechin-3-gallate. Tea is chargeable for abundant qualities that have health benefits including anti-inflammatory, antimicrobial, antioxidative, antitumor, anti-obesity, defence from disorders, and anti-aging activities [39]. The extract of bioactive components obtained from green tea, EGCG, and flavins shows antibacterial activity over *Fusobacterium nucleatum,* pathogenic subgingival known to cause destructive periodontitis. This organism is a typical found to be residing in the human gastrointestinal tract and has been related to inflammatory bowel disease too. Consumption of green tea has hassled protection against the damage caused by these bacteria through leakage of membrane and chelating ions preventing biofilm formation [40].

#### 2.1.1. Fruits and Vegetables

Similar to the skin, it acts as the physical barrier to protect us from the invasion of many pathogens in fruits like the peel outer covering. Several investigation evidences show that the fruit peel is mostly disposed as waste that is found to be sustainable resource containing antimicrobial activity [30, 41]. In a study done by Jagtap and Bapat [42], team has shown pomegranate extract reduces the expansion of *E. coli* due to its great antimicrobial activity as it contains phenols and flavonoids. This study demonstrated similar effect even against other microbes such as *S. aureus and B. cereus* at a degree of 0.01%. In parallel, several other fruits peel such as lemon grass, citrus, and lime peel extract also exhibited antimicrobial and antibacterial activities over products like meat by inhibiting a wide variety of microbe like *S. aureus, E. coli, P. aeruginosa, B. cereus,* and *S. typhimurium* [43]. The antimicrobial activity of peel and capsicum was reported by researchers and was mainly found to be due to the phenolic compounds present in it like the coumaric acid, highly active against *S. typhimurium* and *P. aeruginosa* on minced beef [44]. An organic sulphur compound allicin extracted from garlic has antimicrobial activity on both Gram-positive and Gram-negative bacteria such as *E. coli, Salmonella, Streptococcus, P. aeruginosa, B. cereus, Klebsiella, Helicobacter pylori, Proteus,* and *S. typhimurium* by inhibiting their growth. It is used as preservative and also has health benefits. Aqueous extracts of garlic have been beneficial for their antimicrobial properties such as *S. aureus* in hamburger [45]. The antimicrobial effect of onion extract shows high significance with antibacterial activity against *E. coli,* yeast, and moulds with increased concentrations of the extracts. Antimicrobial efficacy of curcumin, the active metabolite derived from the turmeric plant, has been evaluated against various food pathogens such as *S. typhimurium*, *Listeria monocytogenes, S. aureus*, and *E. coli* showed exceedingly good results in minced meat [46].

The article "Role of Antimicrobial Drug in the Development of Potential Therapeutics" was published in 2022. Journal: Evid Based Complement Alternat Med.

### 2.2. Antimicrobials from Animal Origin

Chitin on partial deacetylation gives chitosan that is a natural polycationic linear polysaccharide obtained basically from the shells of marine crustaceans. Since it has less allergic, nontoxic, and biodegradable, it has been used in wider applications that include antifungal, antimicrobial, antibacterial, and antioxidant activity [47, 48]. It is active against Gram-negative bacteria such as *Bacteroides fragilis, Shigella dysenteriae, E. coli,* and *Vibrio cholerae*. Defensin, a small cationic peptide, has been known for their antibacterial and antimycotic activities [49]. Lysozyme, a polypeptide chain consisting of 129 amino acids, is naturally found in tears, saliva, milk, and breast milk with good antimicrobial activity against bacteria causing death by cleaving glycosidic linkages in the cell wall peptidoglycan. It is a crucial defence mechanism with being taken into account the most important element of the innate immune system in mammals [50]. Avidin, a charged glycoprotein, binds to biotin both present in egg that makes unavailable for the microbial growth, and spoilage has been an important diagnostic tool immunoassay using avidin-biotin system, thus controlling growth of several microbes such as *Klebsiella pneumoniae, E. coli, P aeruginosa*, and *Serratia marcescens*. An antimicrobial peptide, pleurocidin, is incredibly active against Gram-negative and Gram-positive bacteria. Potentially used in food industries due to their varied applications, heat stability, salt tolerant, and other characteristics favour against pathogens like *E. coli, Vibrio parahaemolyticus,* and *L. monocytogenes* [51].

The article "Role of Antimicrobial Drug in the Development of Potential Therapeutics" was published in 2022. Journal: Evid Based Complement Alternat Med.

### 2.3. Antimicrobials from Microbial Origin

Natamycin produced by *Streptomyces natalensis* is used as food preservative and has been effective against yeast and moulds. However, it does not have effective activity against many of the bacterial pathogens due to its antifungal nature. Nowadays, natamycin has been extensively used due to their effectivity in many food processing industries that include various food products such as meat, juices, and dairy products that are either pasteurised or unpasteurised. Reuterin, a water-soluble antimicrobial derivative obtained from *Lactobacillus reuteri*, is a nonproteinaceous substance that has been found to have a very broad antimicrobial activity. Importantly, it has been effective against both Gram-positive and Gram-negative bacteria, filamentous moulds, and nonfilamentous fungal organisms. It has shown a very high effectivity to a wide selection and range of pH and immune to various enzymes that include proteolytic and lipolytic. Most importantly, it exhibits bacteriostatic activity particularly against *Listeria* [52] (Table 2) [53–74].

#### 2.3.1. Prebiotic and Probiotics Mechanism

One of the most important probiotic microbes, lactic acid bacteria (LAB), helps to confer many health benefits and also acts as preservative. These LABs inhibit the expansion of pathogens by the various antimicrobial agents produced by them that includes the organic acids and bacteriocins that are antimicrobial peptides (Table 2). Different strains of bacteria like *L. sakei* and *L. curvatus* are effective against many pathogens like *Escherichia O157:H7* and *L monocytogenes* [75]. Bacteriocins are the antimicrobial compounds that are produced majorly by Gram-positive bacteria, like the LABs, and these metabolites are formed during their growth. These metabolites are polypeptides, wherein the manufacturing microbes gain an advantage to compete with the other microorganisms for their survival [76].

It is well established the advantages of probiotics associated with human health. Mechanisms are possibly being multifactorial, one postulated being antagonistic mechanism on pathogens competing for the nutrients for growth factor, and provide and enhance functions of the gut barrier, competitive adherence to the mucosa and epithelium, defence by the production of antimicrobial substances, and immune system modulation [77, 78]. These probiotic microbes consume most of the monosaccharides in the GI tract making it unavailable for the pathogens such as *Clostridium difficile*. Lysins have also been improved by bioengineering; for instance, a novel chimeric lysin was constructed by combining the active site present on the lysin protein with a cell wall binding domain [78]. Modulation and enhanced gene expression involved by a number of *Lactobacillus spp* like the tight junction signalling of E-cadherin and *β*-catenin has helped to reinforce the integrity of intestinal barrier. Several proteins by these *Lactobacillus spp* promote the mucosal adhesion by displaying surface adhesins and integrate with complex glycoprotein like mucin, secreted by the intestinal epithelial cells to prevent pathogens [77].

The article "Role of Antimicrobial Drug in the Development of Potential Therapeutics" was published in 2022. Journal: Evid Based Complement Alternat Med.

Another mechanism includes modification of microbial flora by the low and high molecular weight compound synthesis like organic acid (acetic and lactic acids) and antimicrobial compounds like bacteriocins [77]. They exhibit strong inhibitory effect by lowering the intracellular pH or accumulating the ionised forms of organic acids that help in disrupting the pH balance and consequently inhibiting growth of pathogens like *Helicobacter pylori* that causes gastrointestinal disorders and cancers. Bacteriocins produced by probiotics, lactacin B from L. acidophilus, bifidocin B produced by *Bifidobacterium bifidum* NCFB 1454, plantaricin from *L. plantarum*, and nisin from *Lactococcus lactis* [79] have antibacterial activity against the food-borne pathogens by destructing the target cells by pore formation or inhibiting cell wall synthesis [80].

### 2.4. Miscellaneous Antimicrobial Agents

Antimicrobials are derived from different sources present either in nature or synthesised through artificial and chemical means. As such, today the antimicrobial drugs are of many diverse types based on their source. Microbe-based antibiotics are the most common types, with penicillin from the various *Penicillium spp* being the first known microbe derived antibiotic to be used by humans. Others include vancomycin derived from *Actinobacteria sps, Amycolatopsis orientalis,* and Streptomycin from *S. griseus*. Plant-based antimicrobials are also another class of antimicrobial agents. These are the beneficial nutrients that we attain from plants that help boost our immunity. Apples are a very good example as they are rich in flavonoids, which have strong antioxidant properties, which are harmful to a large number of microbes [81]. Another well-known is aloe vera, whose latex compound is disruptive towards microbes such as *Corynebacterium*, *Salmonella*, *Streptococcus,* and *S. aureus* [82]. Certain phytochemicals derived from plants have also shown mechanisms to stop microbial proliferation like catechols can cause substrate deprivation in microbes [83], capsaicin initiates membrane disruption [84], and fabatin can form disulphide bridges [85]. Phytochemicals used as antibiotics will majorly contain phenolics and polyphenols that are highly effective against bacteria, fungi, and even viruses. Additionally, they pose significant important group, quinones, which forms complex irreversibly with proteins made of amino acids that are nucleophilic in nature results in their inactivation and loss in the function of proteins [86].

The article "Role of Antimicrobial Drug in the Development of Potential Therapeutics" was published in 2022. Journal: Evid Based Complement Alternat Med.

## 3. Role of CRISPR as an Antimicrobial Agent

Infectious disease continues to pose an enormous burden globally, with the advancement in developing new tools and therapeutics to study the mechanism of host-microbe interactions, and it has not been a tedious job to diagnose and treat infections accurately. Clustered regularly interspaced short palindromic repeats (CRISPR) present in bacteria as well as the members of archaea that act as defence mechanism in protecting them from the invading viruses and bacteriophages. It functions as an adaptive immune system for prokaryotes. It was first discovered in *E. coli* as a homologous repeat of 29 nucleotides separated by 32 nucleotides spacers [87]. It is used for genome editing and evolutionary analysis of prokaryotic strains and has been identified as a major breakthrough mechanism in the field of science and clinical research. It has been known to regulate stress-related phenomenon in bacteria. One of the global threats contributes to a high mortality rate worldwide in spreading infectious diseases. In order to contain the spread of such pandemics, it is highly crucial to get accurate knowledge of the pathogenesis of bacteria, fungi, viruses, and parasites and, further, know the diagnosis and treatments of such diseases. CRISPR and CRISPR-associated proteins have come into the light for their varied applications in the field of infectious disease, evaluation of host-pathogen interaction, development of diagnostic tests, and prevention of such diseases [88]. CRISPR-Cas9 mechanism has been expansively used across various disciplines, like basic sciences, food and crop development, fuel generation, drug development, and human genome engineering [89]. Rapidly emerging multidrug-resistant strains, it has been tough game to combat diseases. The approach of CRISPR-Cas is recognised as a novel means to control multidrug-resistant bacteria. The rise in antibiotic-resistant strains far exceeds than the development of new antibiotics, which has caused a massive rise in the emergence of diseases. CRISPR-Cas system has also been successful in removing resistant microbiome from the gastrointestinal tract, thus reconstructing a healthy and balanced human microbiome. The CRISPR mechanism is quite comparable to that of RNA interference in eukaryotes, wherein small RNA identifies and neutralises specific DNA sequences, later specifically cleaves DNA encoding the antibiotic resistant genes. This includes the following:

- Conjugation-based delivery
- Phage-based delivery
- Nanoparticle (NP)-based delivery
- Antibody-based therapy

The aim of using CRISPR-Cas-mediated methods is to ensure novel ways of developing antibiotics and to combat the MDR pathogens as they use of CRISPR-Cas9 and plasmids to kill bacteria carrying antimicrobial resistance genes (AMR). Alongside, CRISPR-Cas mediated by phages intends to carry plasmids carrying AMR genes leading to the bacterial cell death [90].

The article "Role of Antimicrobial Drug in the Development of Potential Therapeutics" was published in 2022. Journal: Evid Based Complement Alternat Med.

Until date on record, there have been two classes of CRISPR-Cas system, further comprising six subtypes.

  Class 1 CRISPR—Types I, III, and IV—Multiple Cas proteins
  Class 2 CRISPR—Types II, V, and VI—Single Cas protein

CRISPR technology is mainly applied to upregulate or downregulate gene transcription, which is controlled by the activated Cas9 protein through the gene expression. At the molecular level, the genomic locus of CRISPR acts as memory unit wherein the sequences of nucleic acids of the invading pathogens are isolated or hidden away. These particular sequences later help to guide Cas proteins to eliminate the foreign invaders (Figure 2) [91]. Hence, this technology aids to understand regulation of infection causing genes in bacteria, fungi, and viruses. Same knowledge is implicated to combat them by designing accurate therapies and vaccines. The mechanism of CRISPR technology targets nucleic acids upon entry of plasmid DNA or attachment followed by injection of viral genetic material in the host with a progressive step accommodating the Cas gene (Figure 2). When a bacteriophage or plasmid invades a bacterium, a small portion of the DNA that has been invading is cleaved with the help of Cas protein and inserted into CRISPR locus and thus creates memory of sequences [92, 93]. CRISPR ribonucleic acid (crRNA) containing both a single CRISPR and spacer repeat is released into the cytoplasm that manages to bind to the complementary DNA or RNA sequences [94]. Thereafter, a cleavage complex is formed that includes crRNA, its target sequence, Cas nuclease, and a tracer RNA, which cleaves the target at a site adjacent to the crRNA target sequence. As an outcome, this CRISPR-Cas technique has been well contributing in rapid and precise diagnosis of infectious disease. It has allowed enhanced clinical care and manages infection control leading to limited spread of the infection.

The article "Role of Antimicrobial Drug in the Development of Potential Therapeutics" was published in 2022. Journal: Evid Based Complement Alternat Med.

In 2016, Winter and team used CRISPR-Cas single-guide ribonucleic acid (sgRNA) to nullify the effect of haemolysins, a toxin produces by *S. aureus* responsible lysis of red blood cells. Hence, sgRNA can be an efficient tool to elucidate *α*-haemolysin function in *S. aureus* virulence factor that induces cytotoxicity [95]. In addition, around seven genes including EMC2, EMC3, SEL1L, DERL2, UBE2G2, UBE2J1, and HRD1 have been identified and reported to inactivate viral particle responsible for West Nile virus known to cause neuronal cell death [96]. These genes have been an important part of the protein degradation pathway and are part of endoplasmic reticulum that has led to the development of novel drug.

Likewise, CRISPR technology has also been employed to mute toxoplasmosis and Chagas disease initiating protozoal parasites like *Toxoplasma gondii* and *Trypanosoma cruzi*, respectively [97]. This kind of paralysing the protozoal parasite is due to blockade of paraflagellar rod proteins (PFR), which are required for the motility and the attachment of the parasite flagella to the cell host [98]. Pardee et al. [99] performed an experiment that combined nucleic acid sequence-based amplification (NASBA), a process involving isothermal reactions for amplifying RNA along with CRISPR that help to distinguish closely related Zika virus strains. Upon the cleavage of dsDNA with sgRNA-Cas9 complex, either curtailed or full-length DNA fragments are produced. This activated to trigger sequence to NASBA-amplified viral RNA, which caused colour change on the paper disc that enables the strain differentiation.

Centre for disease and control and prevention had reported about 2 million infections were present worldwide and close to 23,000 deaths in the USA every year due to antibiotic resistant bacteria. Keeping this in challenge CRISPR-based technology aims to prepare therapeutics to target not only drug resistant bacteria but also highly infectious viruses such as hepatitis B (HBV) and human immunodeficiency virus (HIV) [100]. One of the applications of CRISPR is to produce selective antimicrobials for annihilating pathogenic bacteria. One example can be selectively killing specific strains of bacteria like *Staphylococcus* and *Escherichia* among pure and mixed cultures by CRISPR-Cas system [101]. Similar practice was also followed by Bikard et al. [102] to selectively kill virulent *S. aureus* strains with the destruction of plasmids in these bacteria carrying mecA methicillin-resistant gene. By contrary, host bacteria with RNA-guided Cas9 protein remained unaffected.

The article "Role of Antimicrobial Drug in the Development of Potential Therapeutics" was published in 2022. Journal: Evid Based Complement Alternat Med.

Nowadays, DNA endonuclease to targeted CRISPR Trans (DETECTR) technique is more frequently being used. It involves the combination of isothermal recombinase polymerase amplification with Cas12a enzymatic activity. This can be used to differentiate between two high-risk strains of human papilloma virus 16 (HPV16) and HPV18. Both are known to cause various types of cancers such as anal, throat, cervical, vaginal, and vulvar mainly in female. A study includes the collection of 25 human anal swab samples followed by testing with DETECTR and PCR analysis. Results showed that all the specimens were correctly identified within an hour of DNA extraction, while the samples that were tested by PCR displayed only twenty-three correctly identified samples signifying the importance of this technique [103].

## 4. Phage-Based Antimicrobial Agents

The rise of MDR strains in recent years is an ongoing struggle in the medical field, due to the ineffectiveness of antibiotics against them. However, to combat this one effective development was the use of bacteriophages as the active antimicrobial agents. Phage therapy has been around for almost a century and used to treat bacterial infections utilising naturally occurring phages. Recent advances have developed the use of bioengineered phages and the specific use of purified lytic proteins isolated from them. Phages exhibit the use of two major protein classes in their action of lysing bacterial host cells.

These two proteins are as follows:

- Transmembrane protein holin
- Peptidoglycan cell hydrolase endolysin

Both mechanisms work combined to bring about bacterial lysis leading to death. The cell membrane pores attach to the holing protein causing an opening to appear, which in turn facilitates lysin protein to gain access cell wall and further hydrolysing it [104]. Phages code for numerous lysin and holing proteins, of which some are very specific, and others are effective in a broad-spectrum. Currently, we identified lysins ABgp46. ABgp46 are highly effective to lyse various strains of Gram-negative strains and MDR strains such as *A. baumanii, P. aeruginosa,* and *S. typhimurium* [105].

Phage lysins have become a topic of interest as they are capable of even lysing bacterial cells by themselves, while holins cannot act alone. Their use in research has been a boon in treating bacteraemia in mice caused by the strains of *A. baumanii* [106], *S. pneumoniae* [107], and methicillin-resistant *S aureus* (MRSA) [108]. Another study showed that uses of phage lysins with antibiotic combinations are found to be more efficient in action against infections as compared to the antibiotics. The study was performed *in vivo* and *ex vitro* in a colon model, with the organism *C. difficile* [109]. The effectiveness of lysins by a recent study showed that they can cross the epithelial cell barrier and affect hard to treat intercellular infections by *S. pyogenes* [110]. Furthermore, they disrupt vegetative cells that were illustrated through the *B. anthracis* lysin PlyG, which exhibited the ability to eliminate endospores of *Bacillus*. Another advantage of phage lysins is that they can be easily produced in large scale through simple recombinant techniques, as demonstrated by the bacteriophage-derived cysteine gene and histidine-dependent amidohydrolase/peptides that are cloned and inserted in *E. coli* where it was then overexpressed for further purification [111]. Lysins have also been optimised through bioengineering; were synthesis of a novel chimeric lysin by using a cell wall binding domain to combine the active site present on the lysin protein. This chimeric lysin has shown the ability to treat MRSA bacteraemia in mice [112].

The article "Role of Antimicrobial Drug in the Development of Potential Therapeutics" was published in 2022. Journal: Evid Based Complement Alternat Med.

## 5. Peptides and Peptide-Related Molecules

Biomolecular recognition in signalling steps in biology leads to the importance of nucleic acids, carbohydrates, or lipids in ligand-target interactions, and the effectors of most signal transduction processes are peptides. Peptides can be of various types that can be fragments of proteins, hormones, cytokines, toxins, and antimicrobials [113]. MDR pathogens have spread rapidly causing nosocomial infections increasing mortality and causing concerns on global health issues [114–116]. With the lack of new antibiotics, the discovery of natural structures has been increased drastically for their role in antimicrobial activity. Antimicrobial peptides (AMPSs) are a part of innate immune defence in all class of life that has gained popularity and has been widely studied for their antimicrobial molecule potential [117]. These bioactive peptides have various biological functions and help in contributing towards human health. They have been variedly used for their therapeutics that include antioxidant, antimicrobial, and antithrombotic effects. Recent years has seen the varied applications of these peptides for disease management, peptide vaccines, and toxicity-related issues.

There is a dilemma for the direct administration of the biopeptides and their derivatives with respect to their *in vivo* stability. However, their therapeutics can be improvised by their coupling with lipids, nonpeptide antibiotics, immunoglobulins, photosensitisers, etc. [118]. Animal models for *Neisseria gonorrhoeae* and *N. meningitidis* were found to be susceptible to 2-pyridone nonapeptide, while the Gram-positive gut bacteria were not affected. DNA biosynthesis inhibition has paved way for bactericidal action and it has been suggested that peptides based on pH activity is actively used against the *Helicobacter pylori* and lipopeptide daptomycin that is been used for treating systemic infections that are caused by MDR Gram-positive bacteria (Figure 3) [119, 120].

The article "Role of Antimicrobial Drug in the Development of Potential Therapeutics" was published in 2022. Journal: Evid Based Complement Alternat Med.

Gram-positive bacteria produce peptides such as lantibiotics that have rare post-translational modified thioether amino acids like lanthionine and methyl-lanthionine that are effective at low nanomolar concentrations and resistance against bacterial proteases. Recently, lanthionine rings made up of nisin (rings D and E) have been identified, which has been cleaved by the nisin resistance protein of *Streptococcus agalactiae*, that can help us in synthesising nonhydrolysable nisin analogues [121]. Furthermore, efforts using bioengineering techniques have made possible to modify these lantibiotics producing genes so that newer variants of them can be discovered [122].

Several marine microbes have been studied, and it has been denoted that about 10 different antibiotic metabolites have been found to be synthesised by them. One such example includes species of *Entotheonella*-producing antibiotic mundticin [123]. Microbes isolated from the gut bacteria of cotton leaf-worm has been fascinating for their production of antimicrobial peptides (AMP), a peptide that helps protect the insect from virulent pathogens. Currently, this has been used as a potential application in microbial coatings and in various food additives [124]. Others include the microbes that are commensals of the human beings like the *Staphylococcus lugdunensis* and *Streptomyces formicae* that produce lugdunin and formicamycins, respectively, and are found to be present in the nasal tract [125, 126].

The emerging multidrug resistance pathogen is one of the biggest threats to human beings with getting treatment options for such infectious disease. *S. salivarius* has been varied studied for its novel bacteriocins that have been a promising antimicrobial activity towards various pathogens. Salivaricins belong to lantibiotics produced by *S. salivarius* that have selective antimicrobial activity against the oral and upper respiratory tract pathogens (Figure 3). In salivaricin, a lantibiotic peptide synthesises molecules of salivaricin (SalA, SalB, Sal9, SalG32, and SalE) that regulate the immune system. In regulatory system, the LanK and LanR proteins represent sensors that check incidence for the Salivaricin active molecules present in the extracellular environment that induces transcription of lantibiotics structural and immunity genes [127–129]. Synthesis of unmodified inactive linear peptide generated is modified by enzyme LanM. LanT protein transports active peptides across the cell membrane. LanFEG, the self-immunity protein, is the form of ABC transporters that helps to expel the active form of lantibiotics from the cell membrane and thus helps to prevent the pore formation and/or disruption in the cell wall synthesis. In case of nisin and other peptides, encoding through clusters for the transport system involves possibly for the self-protection like lanE, LanF, and LanG (Figure 3). These salivaricins have been in limited use as of now for developing probiotic strains of *S. salivarius*-producing molecules that have been studied *in vivo* while colonising the oral cavity. The structure and mechanism of action have been well revised as an important aspect to help enable them in designing newer antimicrobial lantibiotics in the future. Salivaricins are produced by some strains of *S. salivarius* entirely present in human oral cavity, a polycyclic peptide made of lanthionine, and/or *β*-methyllanthionine residual molecules. These molecules stem an important role of having antimicrobial affect towards the relevant oral pathogens that has been utilised for the development of probiotic strains that produce salivaricin. In the future, these molecules might help to prove a greater value for developing novel antimicrobial treatment options in the emerging multidrug resistance pathogenic era [127].

The article "Role of Antimicrobial Drug in the Development of Potential Therapeutics" was published in 2022. Journal: Evid Based Complement Alternat Med.

## 6. Nanoparticles Action as Antimicrobials

In recent years, there is a rapid growth in nanotechnology and has new possibilities opened up for controlling microbial infections by using a variety of NPs as drug delivery systems. Usage of conjugated NPs or green synthesized NPs (GSNPs) is becoming more popular from quite a decade because of the dual activity of metallic NPs added with biological origins boost the activity. Therefore, this synergistic effect may be novel-approaching MDR across pathogenic microbes. Various studies exhibit the strength of NPs as a competent antimicrobial agent, possible antifungal, and feasible antiviral with rich anti-inflammatory properties if it is derived from biological basis. Here, the overall mechanism of the NPs or GSNPs showing boundless antimicrobial activity will be due to denaturation microbial outer membrane leading to fragmentation, inference with disulphide or sulfhydryl bonds, or groups of many enzymes, and interruption with the metabolic processes leads to the death of microbial cell by the generation and liberation of reactive oxygen species (ROS) [130–132]. Intensification of the activity is seen when metal oxides are synthesis using plant because biomolecules of various plant sources exhibit a strong reducing forte as well as act as stabilisers in combination with several classes of flavonoids, proteins, tannins, phenols, and terpenoids accompanied during GSNPs. They are also capable of releasing metal ions that can penetrate into the cell and hinder their metabolic processes [133]. To fulfil this, metal NPs such as copper, silver (Ag), silica (Si), zinc, gold, and copper are extensively used in various fields and it poses superb antimicrobial agents to prevent the pathogens with broad-spectrum activity. Charged NPs help to get adhered on the cell surface helping them to penetrate directly into the cell releasing metal ions; further, ions also destabilise the membrane potential leading to cell leakage. Cell wall destabilisation helps to increase bacterial permeability allowing larger NPs to enter cell to have antibiotic like effect [134].

The article "Role of Antimicrobial Drug in the Development of Potential Therapeutics" was published in 2022. Journal: Evid Based Complement Alternat Med.

Hurdle lays in the microbes specially bacteria-forming biofilms, which make them to secrete strong diverse polysaccharides and cover up facilitating the rapid multiplication of them. This complex aggregates now protect the bacteria and, on the other hand, prevent to diffusion capacity for the antibiotics and hence make the disease or infection more chronic. Hence, these studies have shown that biofilms and drug-resistant bacteria can effectively killed by SiNPs produced by peppermint oil and cinnamaldehyde against *E. coli, P. aeruginosa*, *Enterobacter cloacae,* and *S. aureus* with a removal rate of 99.9% clearance [135]. High concentration of AgNPs is lethal to bacterial cell resulting extreme levels of oxidative stress (inactivation of enzymes and inhibiting bacterial growth) [136, 137]. To evidence this, a study concluded the effective treatment option using AgNPs, which is used for killing chlorine-resistant apicomplexan parasite *Cryptosporidium parvum* [138]. Furthermore, AgNPs showed effective results against HIV1 for the antiretroviral activity and aids as a potent viral inhibitory agent. They are also effective against the HBV [139]. Popularisation of GSNPs in the current situation hires usage of Ag in the production of AgNPs by the extracts of lichens to exhibit tremendous antimicrobial activity. Siddiqi et al. [140] reported lichens such as *Usnea longissimi*, *Xanthoria elegans*, *Cetraria islandica*, *Usnea Antarctica*, and *Leptogium puberulum* yield good amount of AgNPs, which blocks the growth of pathogens such as *S. aureus*, *Streptococcus mutans*, *S. pyogenes*, *S. viridans*, *Corynebacterium diphtheriae*, and *C. xerosis* [141]. AgNPs cannot directly inhibit BSA and PVP as they are completely encapsulated and there is no exposed surface for AgNPs-virus interactions. Hence, foamy carbon AgNPs have comparatively higher surface of display for the virus attachment, which shows higher cytotoxicity to BSA and PVP resulting in the inhibition [142].

The article "Role of Antimicrobial Drug in the Development of Potential Therapeutics" was published in 2022. Journal: Evid Based Complement Alternat Med.

Antimicrobial activities in bacteria and fungi with the use of graphene, graphite graphene oxide, and reduced graphene oxide have been well studied. As graphene (G), NPs gain lot of importance in several carbon-based NPs for multidisciplinary research employed in designing biomedical tools and devices implants, surgical instruments, protein bio-functionalisation, dental accessories, devices used for drug delivery, and many more [143, 144]. The background in this respect has led to the research that GNP derivatives are been found to kill bacteria by membrane disruption and oxidation stress and hence great antimicrobial agent [130–132, 145]. Bactericidal role was detected against *E. coli* and *S. aureus* when being treated with GNPs and found to be useful when used in the dental implants [146, 147]. ZnNPs were used in a study by Khan (2016) that displayed significant good blockade in the growth of bacteria like *E. coli* and *B. subtilis* along with fungus *Candida albicans* [148]. Battery of ZnNPs bactericidal activity is seen across several strains includes *B. cereus, P. aeruginosa*, *S. aureus, K. pneumoniae, Salmonella spp, L. monocytogenes,* and *E. faecium* [149] evincing its broader antimicrobial implications. Considerably, CuNPs have been extensively studied for its antimicrobial activity against *E. coli*, *V. cholera, P. aeruginosa*, *S. typhus*, *S. aureus*, *E. faecalis*, *B. subtilis,* and *S. faecalis* [150]. Cu NPs also have a high antimicrobial effect. They are thought to function against a broad range of bacterial species by interacting with —SH groups and causing proteolysis. These also have a strong affinity for amines and carboxyl groups found on cellular membrane. Cu NPs can disrupt genetic material by linking nucleic acid strands once they penetrate, resulting in bacterial cell death [151]. Low concentration (5 *µ*g/mL) of these CuNPs showed its remedial power by successfully inhibiting the bacteria such as *B. cereus*, *Proteus mirabilis,* and *Aeromonas caviae* [152]. Alavi and team worked with the synthesis of GSNPs using a group of crustose lichen, for example, *Protoparmeliopsis muralis,* with oxide metals like Ag, Cu, Zno, TiO_2_, and Fe_3_O_4_ checked for different activities that include the antiviral, antimicrobial, antibiofilm, antiquorum sensing, and antioxidant agents against the MDR strains of *S. aureus* [153]. This study concluded lichen extract generated NPs showed good result by inhibiting the growth of *S. aureus.* Alongside research has shown that the nanocomposites of Fe_3_O_4_ with SiO_2_ and ZnO/TiO_2_/SiO_2_ have effective antifungal properties against Candida spp., like *C. albicans,* Aspergillus spp., such as *A. flavus, A. Niger, and A. terreus* [154]. In biological system, magnesium oxide (MgO) assists an excellent natural reducing agent, several studies have used for the GSNPs using plant extracts like aloe vera (*A. barbadensis Mill*), Pigeon wings plant (*Clitoria ternatea*), and Indian gooseberry (*Emblica Officinalis*), and the combination of metal oxide and plant extract boosts the antioxidant property and helps to destroy the harmful pathogens. In a recent investigation, GSMgONPs made by using aqueous juice extract of Indian gooseberry (*Phyllanthus emblica*) commonly called as amla displayed exceptional antibacterial activity by obstructing the growth of human pathogens, namely, *P. aeruginosa*, *S. aureus, K. pneumoniae,* and *E. coli* [130]. Therefore, these metal NPs can be extensively helpful in biomedical sciences and engineering with their vast applications that include antibacterial, antifungal, and antiviral to help combat various infectious diseases. Fe_3_O_4_ in its bulk form is considered inert and lack antimicrobial activity. Surprisingly, these materials can be modified to introduce antimicrobial properties when synthesised in nanosize. Interestingly, microbiological assays have been proved that surface modified using Fe_3_O_4_ nanoparticles demonstrates anti-adherent properties and significantly reduces both Gram-positive and Gram-negative bacterial colonisations [155].

The article "Role of Antimicrobial Drug in the Development of Potential Therapeutics" was published in 2022. Journal: Evid Based Complement Alternat Med.

## 7. Nanoparticles for Immunostimulation

NPs as nanomedicines are also a promising approach in immunomodulation, which interact and modify the immune system's activity resulting in immunosuppression or immunostimulation. These modifying effects may have bidirectional action; positive or negative consequences depend on the factors like as composition, size, and surface chemistry, among other NPs [156]. Metals that do not mainly trigger antigen-specific responses or create metal-specific lymphocytes are used to stimulate immune system cells. Many different forms of NPs have been found to create ROS in vitro and in vivo, enhancing immune function and inflammatory responses [157, 158]. Some nanotechnology-based anticancer therapeutics has antitumor qualities in vitro but promotes tumour growth in vivo. Inflammation is a critical immune system response that may be triggered by NPs, as indicated by the production of cytokines and chemokine. The key downstream processes of inflammation have been identified as oxidative stress produced by NPs. In comparison with regular particles, NPs have a vast surface area and significant oxidative capabilities [159]. The immunological imbalance caused by oxidative damage caused by NPs is a major contributor. Pb-based NPs has also been demonstrated to disrupt macrophage-T cell interactions, lowering macrophage capabilities including phagocytosis, cell adhesion, and nitric oxide generation while enhancing antioxidant activity. These reactions might be attributable to Pb's potential to influence the expression of genes linked to innate immunity [160].

## 8. Antibodies as Treatment Options

With the approval of monoclonal antibodies from past three decades, it has been approved by the United States Food and Drug Administration in 1986. The application of antibodies being engineered has dramatically changed the medical treatment options. Currently, with their high specificity and less adverse effects they make a major class of new drugs for treatment. The market for antibodies as therapeutics has increased drastically over the past five years as the bestselling drug for various treatments that include human diseases like cancers, metabolic disorders, and infectious diseases [161]. Kohler and Milstein produced monoclonal antibodies (mAbs) that are efficient molecules used for therapy for targeting reagents [162, 163]. Antibody like palivizumab has been previously administrated for the prevention of serious lower respiratory tract syncytial virus disease in children documented by the European Medicines Agency, 2013 [164]. The second mAb bezlotoxumab authorised in 2017 to be directed for the use against the infectious disease throughout the European economic area that targets *Clostridium difficile* toxin B for the prevention of recurring infection as it risked in adults due to the repeated [164, 165].

## 9. Conclusion

Globally, antibiotic resistance has drastically increased further increasing the health issues and also the economy. Considering very little advancement towards the discovery of novel antibiotics effective against these MDR strains, use of alternative methods could help to resolve the problem. In this grim scenario, every pharmaceutical and scientific community of the world think for alternative treatment modalities, which can improvise their products and cut down the cost. Alternatives can be derived from the natural sources like bioactive compound or secondary metabolites known from many generations coming from plant extracts, and microbial and metal conjugated with bioactive compounds have antimicrobial characteristics. This approach is quite promising and delivers us new class or old class with active variants. The abilities of microbes and plant derivatives can successfully deliver the novel bioactive compounds, which will become useful therapeutic tools. Also, the application of newer molecular tools and techniques will help to contribute for the next generation of antimicrobial compounds and to combat infectious diseases. Comprehensive applications of phytochemical bioactive molecules and microbial-conjugated compounds have marked significant demand and have challenged innovator to think and develop powerful novel bioactive derivatives as an alternative to conventional treatment regime. Accordingly, new biotechnological strategies involving the phage-based therapy, metal oxide-based NPs, GSNPs, or the role of CRISPR have provided access to detect surface active target sites in pathogens and act on them. The need for treating infections would be further enhanced with findings in the structural analysis and molecular docking helping to design the specific antimicrobials with lesser toxicity, high selectivity, and easily biodegradable. Hence, this should be engrossed as the demand for screening of indigenous molecules from different sources, untrapped traditional formulation, and practices across the world reveals the source of them. Reconsidering the facts of these secondary metabolites of biological origin, one should be ready to exploit microbial and plant diversity, with various other techniques to discover novel bioactive molecules or strategies to treat these pathogens that cause life-threatening diseases and to be used as therapeutic tool.

The article "Role of Antimicrobial Drug in the Development of Potential Therapeutics" was published in 2022. Journal: Evid Based Complement Alternat Med.

## Figures and Tables

**Figure 1:** Diagrammatic representation of different target sites for the antimicrobial agent's activity on a bacterial cell. ❶ Alteration in PBP: modified PBP is responsible for the mechanism of action of resistance seen in Gram-positive bacteria as it produces *β*-lactamases. For example, reduction in affinity of *β*-lactam antibiotics is due to the mutation on penicillin-binding protein. ❷ Efflux pumps: antibiotics are exported via the membrane proteins inside the cell and maintain their low-intracellular concentrations by pumping them out before they reach their target. Several unrelated antibiotics such as macrolides, tetracyclines, and fluoroquinolones (FQ) are been pumped by cytoplasmic membrane-associated multidrug transporters contributing in the development of MDR strains. ❸ Inhibitors of DNA replication: inhibition of the bacterial division by preventing enzyme DNA gyrase activity (nicks double-stranded DNA and negative supercoils and reseals) is facilitated by quinolones like FQ. ❹ Altered cell wall precursors: Gram-positive bacteria can be inhibited by glycopeptides like vancomycin or teicoplanin as they are involved suppression cell wall synthesis. ❺ DNA mutated-DNA gyrase and topoisomerase IV: quinolone mechanism of resistance involves modification of two enzymes: DNA gyrase and topoisomerase IV. Replication failure is due to mutations in genes gyrA and parC making FQ unable to bind. ❻ Folic acid metabolism inhibitors: combination of few drugs like sulphonamides and trimethoprim acts on biosynthetic pathway, which shows synergy and a reduced mutation rate for resistance. ❼ Alteration in the 30S subunit or 50S subunit: resistance to drugs that affect protein synthesis, that is, macrolides, tetracycline, and chloramphenicol, bind to 30S ribosomal subunit, whereas chloramphenicol, macrolides, lincosamides, and streptogramin B bind to 50S ribosomal subunit to suppress protein synthesis. ❽ Inhibitors of protein synthesis: tetracyclines offer resistance by inhibiting integrity of ribosomal structure and RNA polymerase mutations conferring resistance to rifampicin. ❾ Antibiotic inactivation by enzymes: *β*-lactamases, aminoglycoside-modifying enzymes, and chloramphenicol acetyltransferases are the three main enzymes that inactivate antibiotics. ❿ Porins: present in the outer membrane. The changed selectivity or decreased in porins stops the antimicrobials to act on the pathogens conferring resistance.

The article "Role of Antimicrobial Drug in the Development of Potential Therapeutics" was published in 2022. Journal: Evid Based Complement Alternat Med.

**Figure 2:** Illustration of the mechanism of action of CRISPR/Cas in a bacterial cell. (a) Entry of genetic material of virus, phage, or plasmid into bacteria. (b) Short segments with genetic information of the invader inserts into CRISPR region. (c) Expression of crRNA in the bacterium. (d) Cleavage of the invading DNA by the formation of a cleavage complex consisting of foreign DNA, crRNA, and Cas9 protein.

**Figure 3:** Role of antimicrobial peptides (AMPs): in general, (a), (b), and (c) Different types of AMPs act on the pathogens by penetrating the bacterial membrane through the porins and blocking various cellular and physiological processes of the cells, eventually leading to the death. (d) Inactivation of enzymes by peptide molecules. (e) Acts as ATPase inhibitor. (f) Induces cell death via interacting with intracellular DNAs and RNAs inducing DNA damage. (g) Cationic AMPs interact with organelles as in fungi such as mitochondria, eventually leading to fungal death. (h) Inhibition of the synthesis of protein and also cell wall. (i) Endocytosis.

**Table 1:** List of various plant compounds used for their antimicrobial properties [37].

Scientific name	Common name	Compound	Antimicrobial activity
Berberis vulgaris	Barberry	Berberine	Bacteria and protozoa
Piper nigrum	Black pepper	Piperine	*Fungi, Lactobacillus, Micrococcus, E. coli,* and *E. faecalis*
Rhamnus purshiana	Cascara sagrada	Tannins	Bacteria, fungi, and viruses
Matricaria chamomilla	Chamomile	Anthemic acid	*M. tuberculosis, S. typhimurium,* and *S. aureus*
Syzygium aromaticum	Clove	Eugenol	Bacteria, fungi, and Trypanosoma cruzi
Vaccinium spp.	Cranberry	Fructose	Bacteria
Eucalyptus globulus	Eucalyptus	Tannin	Bacteria and viruses
Allium sativum	Garlic	Allicin and ajoene	General
Hydrastis canadensis	Goldenseal	Berberine and hydrastine	Bacteria, *Giardia duodenale,* and *Trypanosomes*
Camellia sinensis	Green tea	Catechin	General
Glycyrrhiza glabra	Licorice	Glabrol	*S. aureus* and *M. tuberculosis*
Quercus rubra	Oak	Tannins Quercetin	
Allium cepa	Onion	Allicin	Bacteria and *Candida*
Mahonia aquifolia	Oregon grape	Berberine	*Plasmodium* and *Trypanosomes*
Thymus vulgaris	Thyme	Caffeic acid, Thymol, and Tannins	Viruses, bacteria, and fungi
Curcuma longa	Turmeric	Curcumin	Bacteria and protozoa

The article "Role of Antimicrobial Drug in the Development of Potential Therapeutics" was published in 2022. Journal: Evid Based Complement Alternat Med.

**Table 2:** Representation of various biomolecules derived from bacteria that have different biological activities/applications

Type	Characteristics	Examples	Producer	Mode of action	References
Bacteriocin type I	Lantibiotics	Nisin Z and Q, Enterocin W	*Lactococcus lactis*	Pore formation in the membrane by permeabilisation	[53]
Bacteriocin type II	Non Lantibiotics	Enterocin, Leucocin, Munditicin, Lactococcin Q, and Lactocyclicin Q	*Pediococcus pentosaceus,* *P. Acidilactici,* *L. sakei,* *L. lactis sub sp. Cremoris,* *L. plantarum,* *L. gasseri,* *Enterococcus faecalis, and* *L. garvieae*	Pore formation in the membrane by permeabilisation	[54–57]
Bacteriocin type III	Large peptides	Lysostaphin, Enterolysin A, Helveticin J	*L. crispatus,* *L. helveticus,* *E. faecalis,* *S. simulans biovar,* *Staphylolyticus,* *Enterococcus faecalis,* *and Lactobacillus helveticus*	Disintegration of the cell-wall imbalance in membrane potential initiating ATP efflux	[58–60]
LPS	Peptides	Surfactin, Iturin, Fengycin	*B. subtilis* *B. amyloliquefaciens*	Antifungal, Antimicrobial, Insecticidal, Antimycoplasma, Haemolysis, and Establishment of ion channels in lipid membranes. Acts as bioagents. Immunomodulatory, antitumor enzyme inhibitors, toxins, etc.	[61–63]
Other bioactive compounds		Vinaceuline	*Streptomyces spp*	Antibacterial activity	[64]
		Halocin	*Haloferax mediterranei*	Alter membrane permeability	[65]
		Sulfolobicins	*Sulfolobus islandicus HEN2/2*	Exact mode of action is not known	[66]
		Lactones	*Phomopsis spp*	Active against *A. Niger* *Botrytis cinerea* *Fusarium*	[67]
		Jesterone	Pestalotiopsis jesteri	Active against *Pythium ultimum, Phytophthora citrophthora, Rhizoctonia solani* *Sclerotinia sclerotiorum*	[68]
		Diastaphenazines	*Streptomyces diastaticus* Sub spp. ardesiacus	Antibacterial and antifungal activity	[69]
		Reuterin	*Lactobacillus reuteri*	Antimicrobial	[70, 71]
		Mollemycin A 20	*Streptomyces spp (CMB-M0244)*	Effective against Gram-positive and Gram-negative bacteria, compound shows antimalarial properties	[72]
		Avermectins	*Streptomyces avermitilis*	Onchocerciasis and lymphatic filariasis	[73]
		Cahuitamycins	*Streptomyces gandocaensis*	Functional by inhibiting biofilm formation in Gram-negative *Acinetobacter baumannii*	[74]

The article "Role of Antimicrobial Drug in the Development of Potential Therapeutics" was published in 2022. Journal: Evid Based Complement Alternat Med.

## Data Availability

All data used to support the findings of this study are included within the article.
